The article "Whole-exome sequencing in patients with premature ovarian insufficiency: early detection and early intervention" was published in 2020. Journal: J Ovarian Res.

# Whole-exome sequencing in patients with premature ovarian insufficiency: early detection and early intervention

**DOI:** 10.1186/s13048-020-00716-6

**Published:** 2020-09-22

**Authors:** Hongli Liu, Xiaoli Wei, Yanwei Sha, Wensheng Liu, Haijie Gao, Jin Lin, Youzhu Li, Yaling Tang, Yifeng Wang, Yanlong Wang, Zhiying Su

**Affiliations:** 1 Department of Gynecology, Key Clinical Discipline of Fujian province, Women and Children’s Hospital, School of Medicine, Xiamen University, Xiamen, 361005 Fujian China; 2 School of Pharmaceutical Sciences, Xiamen University, Xiamen, 361005 Fujian China; 3 Department of Reproductive Medicine, Women and Children’s Hospital, School of Medicine, Xiamen University, Xiamen, 361005 Fujian China; 4 Department of Gynecology and Obstetrics, Zhujiang Hospital, Southern Medical University, Guangzhou, 510000 Guangdong China; 5 Reproductive Medicine Center, the First Affiliated Hospital of Xiamen University, Xiamen, 361003 Fujian China; 6 Department of Obstetrics and Gynecology, the First Affiliated Hospital of Xiamen University, Xiamen, 361003 China

**Keywords:** Premature ovarian insufficiency, Pathogenic variants, Whole-exome sequencing, Early intervention, Compliance

## Abstract

**Background:**

The loss of ovarian function in women, referred to as premature ovarian insufficiency (POI), is associated with a series of concomitant diseases. POI is genetically heterogeneous, and in most cases, the etiology is unknown.

**Methods:**

Whole-exome sequencing (WES) was performed on DNA samples obtained from patients with POI, and Sanger sequencing was used to validate the detected potentially pathogenic variants. An in silico analysis was carried out to predict the pathogenicity of the variants.

**Results:**

We recruited 24 patients with POI and identified variants in POI-related genes in 14 patients, including bi-allelic mutations in *DNAH6*, *HFM1*, *EIF2B2*, *BNC*, and *LRPPRC* and heterozygous variants in *BNC1*, *EIF2B4*, *FOXL2*, *MCM9*, *FANCA*, *ATM*, *EIF2B3*, and *GHR*. No variants in the above genes were detected in the WES data obtained from 29 women in a control group without POI. Determining a clear genetic etiology could significantly increase patient compliance with appropriate intervention strategies.

**Conclusions:**

Our study confirmed that POI is a genetically heterogeneous condition and that whole-exome sequencing is a powerful tool for determining its genetic etiology. The results of this study will aid researchers and clinicians in genetic counseling and suggests the potential of WES for the detection of POI and thus early interventions for patients with POI.

## Background

Premature ovarian insufficiency (POI) is defined as amenorrhea before the age of 40 and is characterized by FSH levels greater than 25 IU/L in two measurements for at least 4 weeks [1]. POI is a severe disorder affecting approximately 1% of women of childbearing age worldwide [2]. Genetic defects are a common cause of POI, as has been proven in a large number of studies. Currently, with the development of technology, more than 100 genes have been found to be associated with POI [3–6].

Whole-exome sequencing (WES) is widely used to identify the genetic etiologies of various diseases [7]. However, gynecologists diagnose and treat POI only based on a patient’s symptoms, and genetic methods have not been widely used to identify the genetic causative factors of idiopathic POI. With the significant decrease in the price of WES, it has emerged as a powerful tool with potential for clinical applications in the early detection of POI and timely intervention for patients with POI. Moreover, a clear genetic etiology could significantly improve treatment compliance.

In this study, we performed WES of DNA samples obtained from 24 patients with POI and found variants in POI-related genes in 14 patients. Therefore, it is possible to conduct etiological testing for patients with POI through WES, which could help in the timely intervention of POI.

## Results

### Clinical features of patients with POI

All 24 patients were diagnosed with sporadic POI according to standard criteria (detailed in the Methods section). Based on the physical examination results, none of the patients showed an obvious abnormality in physical development. The ovaries of all patients could be detected by transvaginal color Doppler ultrasound examination. However, all patients had abnormal hormone levels. All patients with POI had a normal 46, XX karyotype. The clinical characteristics of the POI patients are shown in Table 1.

**Table 1:** Clinical and hormonal characteristics of the patients with POI

Case ID	Age (Years)	Menopause age (Years)	BMI (kg/m2)	Primary or secondary amenorrhea	FSH (IU/L)	LH (IU/L)	E2 (pg/mL)	Karyotype	Ovary size (right/ left, mm)	Follicle
POI-1	35	33	25.20	secondary	35.92	16.61	24	46,XX	21*16/22*18	Rare
POI-3	29	27	28.25	secondary	161.18	56.92	21	46,XX	18*11/16*11	Absent
POI-6	30	28	24.14	secondary	73.77	27.56	79	46,XX	19*11/18*12	Absent
POI-7	23	13	23.80	primary	127.54	39.5	34	46,XX	15*10/13*9	Absent
POI-8	25	15	25.71	primary	92.93	43.38	13	46,XX	10*6/11*5	Absent
POI-9	24	18	25.46	secondary	102.8	38.39	20	46,XX	18*9/21*8	Absent
POI-11	32	31	22.31	secondary	48.65	40.24	18	46,XX	19*12/17*15	Rare
POI-12	28	27	25.65	secondary	86.57	35.77	22	46,XX	16*11/15*9	Rare
POI-14	30	28	22.83	secondary	110.38	51.60	16	46,XX	17*14/16*10	Absent
POI-17	25	24	22.86	secondary	55.24	36.83	15	46,XX	20*14/21*17	Rare
POI-18	27	26	27.55	secondary	60.45	50.46	18	46,XX	18*10/17*8	Rare
POI-21	22	14	23.07	primary	107.28	38.55	24	46,XX	11*6/12*5	Absent
POI-23	26	25	25.81	secondary	38.50	24.69	15	46,XX	17*15/16*13	Rare
POI-24	16	13	24.31	primary	49.66	35.52	33	46,XX	10*5/11*4	Absent

Abbreviation: *FSH* Follicle-stimulating hormone, *LH* Luteinizing hormone, *E2* Estradiol

### Whole-exome sequencing analysis of patients with premature ovarian insufficiency

To characterize the genetic pathogenesis of POI, we performed WES of the DNA samples of the 24 POI patients. We retained the variants with a minor allele frequency of less than 1% in the dbSNP, 1000G, ESP6500, and gnomAD databases. The retained variants were filtered according to the selected candidate genes involved in POI. We identified 19 variants in 12 genes, including compound heterozygous variants in *DNAH6*, *HFM1*, *EIF2B2*, *BNC1*, and *LRPPRC* and nine heterozygous variants in *BNC1*, *EIF2B4*, *FOXL2*, *MCM9*, *FANCA*, *ATM*, *EIF2B3*, and *GHR*, from 14 patients (Table 2). None of the above genes were detected in the WES data from 29 women in the control group.

**Table 2:** In silico analysis of variants found by whole-exome sequencing

Case ID	Zygosity	Gene	Ref mRNA No.	Mutation type	Variants	Amino acid change	gnomAD	PolyPhen/SIFT/MutationTaster/CADD/DANN
POI-1	Het.	*DNAH6*	NM_001370.2	missense	c.2407C > A	p.Q803K	0.000004062	B/T/P/T/T
	Het.			missense	c.8680G > A	p.V2894M	0	D/D/D/D/D
POI-3	Het.	*BNC1*	NM_001717.4	missense	c.1724A > T	p.D575V	0.0003	D/T/D/D/D
POI-6	Het.	*HFM1*	NM_001017975.6	missense	c.3100G > A	p.G1034S	0	D/D/D/D/D
	Het.			splice-site	c.1006 + 1G > T	–	0.00000523	−/−/D/D/D
POI-7	Het.	*EIF2B4*	NM_015636.3	missense	c.1397G > A	p.R466Q	0.00007716	D/T/D/D/D
POI-8	Het.	*FOXL2*	NM_023067.4	missense	c.676G > A	p.A226T	0	D/D/P/D/D
POI-9	Het.	*MCM9*	NM_017696.3	missense	c.2488G > A	p.A830T	0.00002173	B/T/P/T/T
POI-11	Het.	*FANCA*	NM_000135.4	missense	c.2340T > G	p.H780Q	0	D/D/P/T/T
POI-12	Het.	*ATM*	NM_000051.4	missense	c.2367C > G	p.N789K	0	B/T/P/T/T
POI-14	Het.	*EIF2B2*	NM_014239.4	missense	c.76G > A	p.G26S	0.000008134	D/T/D/T/D
					c.922G > A	p.V308M	0.000008122	D/D/D/D/D
POI-17	Het.	*EIF2B3*	NM_020365.5	missense	c.389T > C	p.M130T	0.00003656	B/T/D/D/T
POI-18	Het.	*FOXL2*	NM_023067.4	missense	c.118G > C	c.G118C	0.00001754	D/T/P/T/D
POI-21	Het.	*BNC1*	NM_001717.4	missense	c.1703A > T	p.D568V	0.0003	D/T/D/D/D
				missense	c.1574T > C	p.L525P	0.0006	D/D/D/D/D
POI-23	Het.	*GHR*	NM_000163.5	missense	c.282G > A	p.W94X	0	−/−/D/D/T
POI-24	Het.	*LRPPRC*	NM_133259.4	missense	c.7G > T	p.A3S	0.0001	D/D/D/D/D
					c.2965C > T	p.R989C	0.0005	D/D/D/D/D

Abbreviation: *PolyPhen* http://genetics.bwh.harvard.edu/pph2/. D: Probably damaging (> = 0.957), P: possibly damaging (0.453 < =pp2_hdiv<=0.956) B: benign (pp2_hdiv<=0.452), *SIFT* http://sift.bii.a-star.edu.sg/. D: Deleterious (sift<=0.05); T: tolerated (sift> 0.05), *MutationTaster* http://www.mutationtaster.org/. A” (“disease_causing_automatic”); “D” (“disease_causing”); “N” (“polymorphism”); “P” (“polymorphism_automatic”, *CADD* https://cadd.gs.washington.edu/download. D: Damaging; T: Tolerable, *DANN* https://cbcl.ics.uci.edu/public_data/DANN/. D: Damaging; T: Tolerable

Sanger sequencing was performed on samples from a subset of patients (POI-1, 3, and 6–9) and their family members to validate the variants and investigate inheritance. POI-1 harbored two compound heterozygous variants in *DNAH6*, c.2407C > A and c.8680G > A. Her unaffected mother carried the heterozygous variant c.2407C > A, and her father carried the heterozygous variant c.8680G > A, indicating that the two variants in POI-1 were inherited, one each, from her parents (Fig. 1a). Compound heterozygous variants c.3100G > A and c.1006 + 1G > T of *HFM1* were confirmed in POI-6. The heterozygous c.3100G > A variant was identified in her mother, and the heterozygous c.1006 + 1G > T variant was identified in her father (Fig. 1c). Heterozygous variants c.1724A > T in *BNC1* (Fig. 1b), c.1397G > A in *EIF2B4* (Fig. 1d), c.676G > A in *FOXL2* (Fig. 1e), and c.2488G > A in *MCM9* (Fig. 1f) were identified in POI patients and their fathers. Moreover, as expected, the mothers of these four patients harbored wild-type alleles.

**Fig. 1:** Sanger sequencing validated the POI-related variants. **a** Sanger sequencing validated the compound heterozygous variants of *DNAH6* c.2407C > A and c.8680G > A in POI-1. Her unaffected mother carries the heterozygous variant c.2407C > A, and her father carries the heterozygous variant c.8680G > A. **b** Sanger sequencing confirmed that POI-3 and her father both carry the heterozygous variant c.1724A > T in *BNC1*. **c** Two heterozygous variants, c.3100G > A and c.1006 + 1G > T, of *HFM1* were confirmed in POI-6. Heterozygous variant c.3100G > A was inherited from her, mother and heterozygous variant c.1006 + 1G > T was inherited from her father. **d** Sanger sequencing confirmed that both POI-7 and her father carry the heterozygous variant c.1397G > A in *EIF2B4*. **e** Sanger sequencing confirmed that POI-8 and her father carry the heterozygous variant c.676G > A in *FOXL2*. **f** Sanger sequencing confirmed that POI-3 and her father carry the heterozygous variant c.2488G > A in *MCM9*

### Analysis of the novel variants identified in patients with POI

We evaluated the 19 variants by *in-silico* analysis. First, we assessed the frequency of the variants. Data from the gnomAD database, a rich and informative database containing exome data from the ExAc and 1000G databases, in addition to data from many other databases, suggest that all of these variants were rare, and six of them were not present in the database. These results indicate that the frequency of these variants in the population is extremely low, which is compatible with the incidence of POI. Moreover, 16 of the 19 variants were predicted to be deleterious by five prediction tools, Polyphen-2, SIFT, MutationTaster, CADD, and DANN (Table 2).

## Discussion

In this study, we performed WES of the DNA samples of 24 POI patients and identified pathogenic variants associated with POI in 14 of the patients. Our study further supports the notion that genetic variants of several genes are important in the pathogenesis of POI and may be the main reason for sporadic cases of unknown etiology.

Previous studies have shown that dynein axonemal heavy chain 6 (DNAH6) is involved in generating the force required for ciliary beating, and mutations in this gene may cause primary ciliary dyskinesia, non-obstructive azoospermia, or sperm morphological defects [8–11]. By using a high-resolution array comparative genomic hybridization platform, a 171 kb deletion in *DNAH6* was identified as the main etiology of POI in a patient [12]. POI-1 harbored two compound heterozygous *DNAH6* variants, c.2407C > A and c.8680G > A. Therefore, *DNAH6* is an attractive candidate pathogenic gene for POI.

Basonuclin 1 (BNC1), a zinc finger protein, is abundant in the germ cells of the testis and ovary. BNC1 plays a regulatory role in rRNA transcription during mouse oogenesis, and deletion of the gene (*BNC1*) that expresses BNC1 protein in mice leads to female subfertility, suggesting that BNC1 is essential for oogenesis [13–15]. Haploinsufficiency of *BNC1* has been reported as an etiology of human autosomal dominant POI [16]. Another study found a 1597.8 kb deletion in *BNC1* in a patient with POI [17]. POI-3 carried the heterozygous *BNC1* variant c.1724A > T, and POI-21 carried the biallelic *BNC1*variants c.1703A > T and c.1574 T > C. All three variants were predicted to be disease-causing substitutions. In general, both heterozygous and complex heterozygous mutations in *BNC1* are pathogenic factors for POI, so it is important to pay particular attention to haploinsufficiency caused by heterozygous mutations.

Helicase for meiosis 1 (HFM1) is an ATP-dependent DNA helicase that is mainly expressed in germ-line cells. Defects in the gene *HFM1* cause premature ovarian failure [18–21]. POI-6 harbored the compound heterozygous variants c.3100G > A and c.1006 + 1G > T. Both variants were rare and were predicted to be disease causing. Thus, we suspected that these variants are the main pathogenic determinants in POI-6.

Eukaryotic translation initiation factor 2B (eIF2B), a multi-subunit protein comprising two sets of α, β, γ, δ, and ε subunits, is a guanine nucleotide exchange factor (GEF) specific for eIF2 and a key regulator of mRNA translation. EIF2B2, EIF2B3, and EIF2B4 are the β, γ, and δ subunits of EIF2B, respectively. All three participate in protein synthesis and exchange GDP and GTP for activation and deactivation [22]. Compound heterozygous variants in *EIF2B2* have been identified as a cause of POI in one of four patients by next-generation sequencing [23]. The c.1117C > T (p.Arg373Cys) variant in *EIF2B4* was shown to be associated with premature ovarian failure in two patients at the ages of 13 and 18 years, respectively [24, 25]. POI-14 carried bi-allelic c.76G > A and c.922G > A *EIF2B2* variants. POI-17 carried a heterozygous *EIF2B3* variant, c.389 T > C, and POI-7 carried the *EIF2B4* heterozygous variant c.1397G > A. In women of childbearing age with mutations in eIF2B family genes, special attention should be paid to the possibility of POI.

Leucine-rich pentatricopeptide repeat containing (LRPPRC) protein is a leucine-rich protein with a number of pentatricopeptide repeats. This protein plays multiple roles in cytoskeletal organization, vesicular transport, and transcriptional regulation of both nuclear and mitochondrial genes [26]. Mutations in *LRPPRC* are associated with the French-Canadian type of Leigh syndrome. Surviving females exhibit premature ovarian failure, absent or arrested breast development, a lack of menarche, high follicle-stimulating hormone level, a prepubertal uterus, and small ovaries [27]. POI-24 carried c.7G > T and c.2965C > T bi-allelic mutations in *LRPPRC* and suffered from primary amenorrhea.

Forkhead box L2 (FOXL2, OMIM: 605597) is a forkhead transcription factor that contains a fork-head DNA-binding domain and plays a role in ovarian development and function [28, 29]. Mutations in *FOXL2* are known to cause autosomal dominant POI [30–34]. POI-8 harbored a novel heterozygous c.676G > A variant in *FOXL2*, which has not been reported previously.

MCM9 is a member of the mini-chromosome maintenance (MCM) protein family, which is essential for the initiation of eukaryotic genome replication and renewal of germ-line stem cells [35]. Bi-allelic mutations in *MCM9* cause POI in an autosomal recessive manner [36–38]. Heterozygous variants of *MCM9* cause haploinsufficiency and contribute to the pathogenesis of POI, especially secondary amenorrhea [39]. POI-9 carried a heterozygous *MCM9* variant, c.2488G > A, and suffered from secondary amenorrhea.

FANCA is a Fanconi anemia complementation group (FANC) protein. Two heterozygous variants in *FANCA* were identified in two unrelated POI patients from a group of 50 Han Chinese patients with POI by WES [40]. These heterozygous variants reduced FANCA expression levels*,* and *Fanca*^*+/−*^ female mice showed decreased numbers of follicles with aging [40]. POI-11, who carried a heterozygous c.2340 T > G variant in *FANCA*, was married at 30 years of age and had secondary amenorrhea and POI when trying to conceive.

ATM is a serine/threonine kinase belonging to the PI3/PI4-kinase family. It is a cell cycle checkpoint kinase that plays a crucial role in cell cycle checkpoint signaling pathways, which are required for the cellular response to DNA damage and genome stability [41]. ATM is involved in ovarian function, and ATM deficiency can induce premature ovarian failure [42]. The gonads of patients with *ATM* defects are hypoplastic with germ cell deficiencies [43]. Deletion of the *atm* locus in mice accelerated primordial follicle degradation at prophase of meiosis I during oogenesis, leading to primordial and maturing follicles and oocyte deficiency [44]. POI-12 carried the heterozygous *ATM* variant c.2367C > G and had secondary amenorrhea and POI.

Growth hormone receptor (GHR) is a transmembrane receptor for growth hormone. It binds to GH and undergoes conformational changes, which eventually result in activation of the JAK2/STAT-5/IGF-I signaling pathway [45]. The litter size of *GHR*-knockout mice was significantly reduced due to ovarian defects [46]. POI-23 carried a heterozygous *GHR* variant, c.282G > A, and had secondary amenorrhea. We predicted that the ovarian function of this patient was affected by haploinsufficiency.

WES is an unbiased genetic approach that has advantages for identifying the genetic etiologies of POI in patients without obvious somatic anomalies [47–50]. In addition to identifying the genetic pathogenesis of patients with unexplained POI, WES also shows broad potential for applications in the screening and early diagnosis of patients with POI. POI patients suffer both mentally and physically due to poor treatment outcomes and unclear etiologies. Clear genetic etiologies will allow us to develop more effective treatment strategies and significantly improve patient compliance.

POI has major impacts on the reproductive ability and physical and mental health of affected patients. Hormone replacement therapy can partially relieve the symptoms induced by POI. However, there are limited effective treatments for the associated impaired reproductive capacity. Therefore, it is important to recognize POI in patients as early as possible to establish a fertility reserve (e.g., oocyte cryopreservation). With the significant decrease in the price and comprehensive spectrum of pathogenic genes, WES has good potential for application in the early detection and intervention of POI.

## Conclusions

In summary, we recruited 24 patients with POI and identified pathogenic variants in 14 of these patients. In approximately 60% (14/24) of the sporadic cases in our study, we were able to identify potentially pathogenic mutations, which shows the utility of WES for determining the genetic pathogenesis of POI. Our research showed that WES is an effective method for identifying the genetic etiology in patients with idiopathic POI, which may offer a theoretical basis for the early detection and intervention in patients with potential idiopathic POI in the future.

## Methods

### Patients and control subjects

We recruited 24 patients with POI for this study. POI was diagnosed if a patient had amenorrhea for at least 4 months under the age of 40 years and two consecutive follicle stimulating hormone (FSH) measurements > 25 IU/L taken 4 weeks apart [1]. Patients who had significant POI-related risk factors were excluded, including karyotype abnormalities, autoimmune disorders, a history of radiotherapy, chemotherapy, or pelvic surgery, and so on. After the patients provided written informed consent, we performed WES on DNA isolated from the peripheral blood samples of the POI patients to identify any disease-associated variants. All procedures involving human participants were performed in accordance with the standards of the Ethics Committee of the Women and Children’s Hospital of Xiamen University, Zhujiang Hospital of Southern Medical University, and the First Affiliated Hospital of Xiamen University, and in accordance with the 1964 Declaration of Helsinki and its later amendments or comparable ethical standards. Written informed consent was obtained from each study participant.

### Hormone measurements

Blood hormone (FSH, LH, and E2) levels were measured using a UniCel DxI 800 immunochemistry analyzer (Beckman Coulter Inc., USA) according to the manufacturer’s instructions and requirements.

### WES analysis and sanger sequencing validation

WES was performed as described elsewhere. Variants fulfilling the following criteria were retained: (a) missense, nonsense, frameshift, or splice site variants; (b) allele frequencies < 1% in the dbSNP (http://www.ncbi.nlm.nih.gov/snp/), 1000 Genomes (http://browser.1000genomes.org/index.html), ESP6500 (http://evs.gs.washington.edu/EVS/), and Genome Aggregation Database (gnomAD, http://gnomad.broadinstitute.org/) databases. Sanger sequencing was used to validate the variants found in the WES analysis of the patients and their families.

## Data Availability

The data underlying the findings of this article will be shared on reasonable request to the corresponding author.

## Abbreviations

POI: Premature ovarian insufficiency
WES: Whole-exome sequencing
FSH: Follicle-stimulating hormone
LH: Luteinizing hormone
E2: Estradiol
gnomAD: Genome aggregation database
PolyPhen-2: Polymorphism Phenotyping v2
SIFT: Sorting Intolerant From Tolerant
CADD: Combined Annotation Dependent Depletion
DANN: Domain-Adversarial Training of Neural Networks
